# Face Coding Is Bilateral in the Female Brain

**DOI:** 10.1371/journal.pone.0011242

**Published:** 2010-06-21

**Authors:** Alice Mado Proverbio, Federica Riva, Eleonora Martin, Alberto Zani

**Affiliations:** 1 Department of Psychology, University of Milano-Bicocca, Milan, Italy; 2 Institute of Bioimaging and Molecular Physiology, National Research Council (CNR), Milano-Segrate, Italy; University of Minnesota, United States of America

## Abstract

**Background:**

It is currently believed that face processing predominantly activates the right hemisphere in humans, but available literature is very inconsistent.

**Methodology/Principal Findings:**

In this study, ERPs were recorded in 50 right-handed women and men in response to 390 faces (of different age and sex), and 130 technological objects. Results showed no sex difference in the amplitude of N170 to objects; a much larger face-specific response over the right hemisphere in men, and a bilateral response in women; a lack of face-age coding effect over the left hemisphere in men, with no differences in N170 to faces as a function of age; a significant bilateral face-age coding effect in women.

**Conclusions/Significance:**

LORETA reconstruction showed a significant left and right asymmetry in the activation of the fusiform gyrus (BA19), in women and men, respectively. The present data reveal a lesser degree of lateralization of brain functions related to face coding in women than men. In this light, they may provide an explanation of the inconsistencies in the available literature concerning the asymmetric activity of left and right occipito-temporal cortices devoted to face perception during processing of face identity, structure, familiarity or affective content.

## Introduction

It is believed that face processing involves the activation of the face fusiform area [1] (FFA) mediating the analysis of face structure, the superior temporal sulcus mediating the analysis of eye gaze and facial expressions [2] and the inferior occipital gyrus, being particularly responsive to face parts [3]. Some researchers suggest that face processing predominantly activates the right hemisphere [1], whereas others hold that face processing involves both left and right FFA [4] although each may contribute in a different way [5]. It was hypothesized that left FFA is involved in unfamiliar face coding, whereas right FFA would recognize familiar faces [6]. In another study [7] it was found that FFA lateralization depended on handedness: FFA activation was right lateralized in right-handers but not in left-handers (24/32 participants were females). Rhodes et al., [8] found that both left and right FFAs were activated more strongly to faces than to objects while the total volume of activation was significantly larger in the right than the left hemisphere. However, in a recent fMRI study performed only in women [9] they found a clearly bilateral activation of FG in emotional face processing. Overall, the literature is highly inconsistent about FFA hemispheric lateralization [10] [11], [12] since virtually no neuroimaging study has ever considered viewer's sex.

Electromagnetic recordings have identified a posterior negative response peaking at about 170 ms (N170) that is larger to faces than other visual objects over the right hemisphere, and thought to reflect processes involved in the structural encoding of faces. The combination of electromagnetic and neuroimaging data identified the N1 generator in the ventral occipito-temporal cortex [13]–[16], suggesting that N1 might be the manifestation of FFA activity [17]. A closer examination of the literature shows that face-specific N170 topographic distribution is often but not always right-sided in right-handed individuals. It is of great interest that N170 response was found to be bilateral or even left-sided in studies involving a sample in which women were the majority [18] [19] [20] [21] [22]. The study's aim was to investigate whether there are sex-related hemispheric asymmetries for face processing. Face-sensitive N1 responses were measured over the occipital/temporal cortices in 50 right-handed observers. In two previous studies [23], [24] we found a bilateral activation of occipito/temporal cortex in women and right–lateralized activation in men during infant face processing as indexed by sensory ERP responses. Since in those studies all stimuli were infant faces, it lacked a control condition with non-face objects. We devised a paradigm in which face processing of persons of various age was contrasted with that of technological objects.

## Methods

### Participants

Fifty healthy right-handed Italian University students (25 males and 25 females) were recruited as volunteers for this experiment. They earned academic credits for their participation. All students were matched for educational level across sexes. Their mean age was 22.36 years (men = 23, women = 21.77). All had normal or corrected-to-normal vision and reported no history of neurological illness or drug abuse. Their handedness was assessed by the Italian version of the Edinburgh Handedness Inventory, a laterality preference questionnaire reporting right-handedness (0.80) and right ocular dominance for all participants. An ANOVA on laterality quotients proved no sex difference in the degree of lateral preference between men (0.81, SE = 0.03) and women (0.79, SE = 0.03). Almost half of the women practiced contraceptive control (N = 11). About half women were in the pre-ovulatory phase (N = 12), the others in the post-ovulatory phase (N = 11) at the time of EEG recording. 2 women did not provide data. Experiments were conducted with the understanding and the written consent of each participant. The experimental protocol was approved by the ethical committee of the University of Milano-Bicocca. Data from all participants were included in data analysis.

### Stimuli

Stimulus set comprised 520 colour pictures depicting nice-looking male and female faces of various ages (130 adults of 20–50 ys., 130 children of 7–11 ys., 130 toddlers of 1–2 ys.) and 130 technologic/electronic complex objects of similar size and spatial distribution (see Fig. 1). Attractive faces were used to avoid possible subjective differences in aesthetic appreciation of faces, leading to differences in ERP amplitudes [25]. Possibly gender-biased objects (such as electric iron or shaver) were not included. Faces included neck and the upper portion of chest. Normal proportions between infants and adults were maintained to preserve authenticity of perceptual experience. Eyes were aligned to fixation point. Except for the toddler category (sometimes sex was indistinguishable), all faces depicted an equal number of females and males. All people were smiling or showing a positive facial expression. Positive expressions were used since they are more interesting and are likely to generate greater evoked potentials than neutral expressions [24]. On the other hand, negative expressions were avoided since they are known to strongly activate emotion-related brain regions [26], therefore leading to possible sex differences in brain activation. Faces and objects were presented randomly mixed with 44 equiluminant infrequent targets depicting common natural or urban landscapes without visible persons (e.g., streets, offices, countryside, seascape, etc.). Stimulus size was 7° 9′ 56″×8° 23′ 1″, and average luminance was 16.2 cd/cm2. An ANOVA showed no difference in stimulus luminance as a function of stimulus type (faces: adults  = 16.4; children  = 15.6; toddlers  = 16.7. Objects = 16 cd/cm2;). Each slide was presented for 800 ms at the centre of a PC screen with an ISI ranging from 1300 to 1500 ms. The outer background was dark grey.

**Figure 1:** Exemplars of pictures used as stimuli, depicting female and male faces of 3 different age classes, and technological objects as control stimuli.

### Task and procedure

In order to keep subject's attention toward visual stimulation, the task consisted of responding as accurately and quickly as possible to photos displaying landscapes (urban or natural scenarios without visible persons) by pressing a response key with the index finger of the left or right hand while ignoring all other pictures. The two hands were used alternately during the recording session. The order of the hand and task conditions was counterbalanced across subjects. Participants were comfortably seated in a darkened, acoustically and electrically shielded test area. They faced a high-resolution VGA computer screen located 80 cm from their eyes. They were instructed to gaze at the centre of the screen, where a small circle served as fixation point, and to avoid any eye or body movements during the recording session. Stimuli were presented at the centre of the screen, randomly mixed in 8 different short runs lasting about 2 minutes and a half. For each experimental run target stimuli varied between 4–7. Sequence presentation order differed across subjects.

### EEG recording and analysis

The EEG was continuously recorded from 128 scalp sites at a sampling rate of 512 Hz. Horizontal and vertical eye movements were also recorded. Linked ears served as the reference lead. The EEG and electro-oculogram (EOG) were amplified with a half-amplitude band pass of 0.016–100 Hz. Electrode impedance was kept below 5 kΩ. EEG epochs were synchronized with the onset of stimuli presentation. Computerized artifact rejection was performed before averaging to discard epochs in which eye movements, blinks, excessive muscle potentials or amplifier blocking occurred. The artifact rejection criterion was peak-to-peak amplitude exceeding 50 µV, and the rejection rate was ∼5%. ERPs were averaged off-line from −100 ms before to 1000 ms after stimulus onset. ERP components were identified and measured, with reference to the average baseline voltage over the interval from −100 ms to 0 ms, at sites and latency where they reached their maximum amplitude.

The peak amplitude of occipito/temporal N170 component was measured at P9 and P10 in the time window 140–195 ms. ERP data were subjected to multifactorial repeated-measures ANOVA with one factor between (sex: males, females) and 2 factors within groups. The within factors were: stimulus content (ADULTS, CHILDREN, TODDLERS, OBJECTS), and hemisphere (left, right) for ERP data. Multiple comparisons of means were done by post-hoc Tukey tests.

Topographical voltage maps of ERPs were made by plotting colour-coded isopotentials obtained by interpolating voltage values between scalp electrodes at specific latencies. *Low Resolution Electromagnetic Tomography* (LORETA) was performed on ERP waveforms at n170 time latency. LORETA, which is a discrete linear solution to the inverse EEG problem, corresponds to the 3D distribution of neuronal electric activity that has maximum similarity (i.e. maximum synchronization), in terms of orientation and strength, between neighboring neuronal populations (represented by adjacent voxels). In this study an improved version of standardized weighted low-resolution brain electromagnetic tomography (sLORETA) was used, which incorporates a singular value decomposition-based lead field weighting: swLORETA [27]. Source space properties were: grid spacing (the distance between two calculation points)  = 5 point; estimated signal to noise ratio (SNR, which defines the regularization; a higher value for SNR means less regularization and less blurred results) was 3. LORETA was performed on group data and it identified statistical significant electromagnetic dipoles (p<0.05), the larger the magnitude, the more significant the activation.

A realistic boundary element model (BEM) was derived from a T1 weighted 3D MRI data set by segmentation of the brain tissue. The BEM model consisted of one homogenic compartment made up of 3446 vertices and 6888 triangles. The head model was used for intra-cranial localization of surface potentials. Segmentation and head model generation were performed using the ASA [28].

## Results

Fig. 2 shows grand-average waveforms recorded at occipito/temporal electrode sites as a function of the viewer's gender and stimulus content. Strong gender differences are visible, especially in the degree of N170 lateralization and discriminative response.

**Figure 2:** Grand-average ERP waveforms (N = 50) recorded in men and women as a function of stimulus type over left and right occipito/temporal electro sites. On the right a graphic shows N170 peak amplitude values recorded in response to the 4 stimulus types.

The ANOVA performed on the peak amplitude values of N170 revealed a significant effect of stimulus content (F3,144 = 90.4; p<0.000001), showing a larger response to childish (toddler = −3.95 µV, SE = 0.37; child = −3.44 µV) than adult faces (−2.7 µV, SE = 0.33), as proved by post-hoc comparisons (p<0.01). Furthermore, N170 to faces was much larger (p<0.01) than to objects (−0.32 µV, SE 0.26). The further significance of hemisphere x sex (F1,48 = 7.57; p<0.008) showed the presence of a sex difference in N170 lateralization, with larger N170 over the right (−2.92 µV, SE = 0.55) than the left hemisphere in men (−1.95 µV, SE = 0.42), as indicated by post-hoc tests (p<0.01), and no significant asymmetry in women (RH = −2.35 µV, SE = 0.55, LH = −3.21 µV, SE = 0.42).

ANOVA yielded the significance of stimulus content x hemisphere x sex (F 3,144 = 3.51, p<0.018). Post-hoc tests revealed no sex difference in the amplitude of N170 to objects. Furthermore, they showed a much larger face-specific response over the right than left hemisphere (Tod-obj = 5.4 µV at P10 and 2.41 at P9) in men (p<0.01), and a bilateral face specific response in women (Tod-obj = 3.79 µV at P10 and 3.0 µV at P9). It was also found a lack of face coding effect over the left hemisphere in men, with no difference in N170 to faces as a function of person's age. Conversely, a significant age-coding effect of over both hemispheres was found in women, with a larger N170 to toddler than adult faces (p<0.01) at both P9 and P10 sites and no hemispheric difference in the amplitude of N170 to faces. On the other hand, results showed larger right than left hemispheric responses to faces in men (adults, p<0.04; toddlers and children, p<0.00001). The latter effect is visible in topographical maps of Fig. 3, computed for N170 surface voltages recorded in response to adult faces, separately for men and women.

**Figure 3:** Isocolour voltage topographical maps (left and right side views) showing N170 scalp distribution in female and male observers. N170 response is relative to adult face processing. The time window corresponds to its peak (150–170 ms) of maximum activation.

In order to locate the possible neural circuits subtending face coding in the two sexes, two different swLORETA source reconstructions were performed, separately for men and women, on 170 amplitude measured in the time window 135–185 ms, which are displayed in Fig. 4. The inverse solution showed that the processing of adult faces in women was associated with a significant activity in the left fusiform gyrus (possibly corresponding to FFA), left MOG, right cuneus (BA18), left posterior cingulate cortex, and anterior brain regions (BA10/11), as listed in Table 1. In men processing of adult face was associated with activation in the right fusiform gyrus, the left MOG, right posterior cingulate cortex and anterior brain areas (BA10/11).

**Figure 4:** SwLORETA inverse solution performed on brain activity recorded during the 135–175 ms time window in response to adult faces in the two sexes.

**Table 1:** Tailarach coordinates corresponding to the intracranial generators explaining N170 surface voltage to adult faces in the 135–175 ms time window, according to swLORETA.

Magn.	T-x [mm]	T-y [mm]	T-z [mm]	HEM	Lobe	Area
**WOMEN**						
19.2	−28.5	−76.2	−11.7	L	O	Fusiform Gyrus, BA19
18.9	−38.5	−78.2	3.8	L	O	Middle Occipital Gyrus, BA19
19.6	−18.5	−68	4.7	L	Limbic	Posterior Cingulate, BA30
19.5	11.3	−69	13.6	R	O	Cuneus, BA18
5.81	1.5	38.2	−17.9	R	F	Medial Frontal Gyrus, BA11
**MEN**						
15.0	50.8	−66.1	−10.9	R	T	Fusiform Gyrus, BA19
13.5	−48.5	−77.2	−4.2	L	O	Middle Occipital Gyrus, BA19
13.1	21.2	−68	4.7	R	Limbic	Posterior Cingulate, BA30
3.07	−8.5	57.3	−9	L	F	Superior Frontal Gyrus, BA10

Grid spacing  = 5 mm, estimated SNR  = 3. Power RMS: Women  = 65.9; men  = 45.5.

## Discussion

Overall, electrophysiological and source localization data support previous literature about the existence of specific neural populations in the fusiform area (FG)[1] [2] and the middle occipital area devoted to face processing, as reflected by the amplitude of occipito/temporal N170 component of ERPs. Moreover, they seem to suggest a less marked lateralization in the activity of face-devoted brain regions in women than men. This finding, supported by the presence of a stronger left FG generator in women and right FG generator in men, results in a asymmetrical N170 surface amplitude in men, and a bilateral distribution in women (tending toward the left asymmetry). Moreover, over the left hemisphere N170 amplitude did not vary as a function of face age in men but only in women. And indeed N170 was of greater amplitude to toddlers' than adults' faces in both hemispheres of the female brain. This age coding effect might be due to a series of factor including a bias toward baby schema, for which toddlers' faces are judged as cuter and more attractive than adult faces [29], and have greater attention capturing effects, as well as to more perceptual face-specific mechanisms related to the fact that toddler's faces are more alike (perceptually similar) than adult faces. The sex difference in hemispheric asymmetry finding agrees with Glocker and coworkers's [30] evidence of a clear left FFA activation in women during processing of infant faces. On the other hand, they do not directly agree with a recent investigation [7] suggesting a relation between handedness and FFA lateralization, since our female participants, showing a bilateral response of face responsive areas, were indeed right-handed.

Overall, our results are in line with many studies that show differences between men and women in the degree of lateralization of cognitive and affective processes. Substantial data support greater hemispheric lateralization in men than women for linguistic tasks [31] and for spatial tasks [32]. Gender differences have also been found in the lateralization of visual-spatial processes such as object construction and mental rotation tasks [33], in which males are typically right hemisphere (RH) dominant and females bilaterally distributed. More relevant to the present experiment are the data provided by Bourne [34], who examined the lateralization of processing positive facial emotion in a group of 276 right-handed individuals. Subjects were asked to observe a series of chimeric faces with contrasting expressions and to decide which face they thought looked happier. The results showed that males were more strongly lateralized than women, showing a stronger perceptual asymmetry in favour of the left visual field (RH). There are also a number of studies that have found different degrees of lateralization in the cerebral response of men and women to emotional stimuli: men tend to demonstrate an asymmetric functioning, and women a bilateral functioning [35]–[38]. Notwithstanding the existing supporting literature (including sex differences in lateralized amygdala activity during happy and fearful face perception, e.g. [39]), is certainly not a shared knowledge in cognitive neuroscience that face processing is bilateral in the female brain and right-sided in the male brain, and such an assumption is not made anywhere in cognitive neuroscience manuals or clinical essays on prosopagnosia. For this reason, we feel that the present findings may make a great contribution toward the overall understanding of how faces are processed in the female and male brain in humans.

### Conclusions

The present data reveal a lesser degree of lateralization of brain functions related to face coding in women than men, both in terms of face-related N170 amplitude, and N170 object/face and adult/toddler discriminative response. In this light, our data may also provide an explanation of the inconsistencies in the available literature concerning the asymmetric activity of left and right occipito-temporal cortices devoted to face perception during processing of face identity, structure, familiarity or affective content.
